# Angiopoietin-Like 4 Confers Resistance to Hypoxia/Serum Deprivation-Induced Apoptosis through PI3K/Akt and ERK1/2 Signaling Pathways in Mesenchymal Stem Cells

**DOI:** 10.1371/journal.pone.0085808

**Published:** 2014-01-21

**Authors:** Meng Hou, Jinjin Cui, Jingjin Liu, Fang Liu, Rui Jiang, Kai Liu, Yongshun Wang, Li Yin, Wenhua Liu, Bo Yu

**Affiliations:** 1 Key Laboratories of Education Ministry for Myocardial Ischemia Mechanism and Treatment, Harbin, Province Heilongjiang, China; 2 Department of Cardiology, The Second Affiliated Hospital of Harbin Medical University, Harbin, Province Heilongjiang, China; 3 Intensive Care Unit (ICU) Department, The Second Affiliated Hospital of Harbin Medical University, Harbin, Province Heilongjiang, China; Seoul National University, Republic of Korea

## Abstract

Angiopoietin-like 4 (ANGPTL4) is a potential anti-apoptotic agent for various cells. We examined the protective effect of ANGPTL4 on hypoxia/serum deprivation (SD)-induced apoptosis of MSCs, as well as the possible mechanisms. MSCs were obtained from rat bone marrow and cultured *in vitro*. Apoptosis was induced by hypoxia/SD for up to 24 hr, and assessed by flow cytometry and TUNEL assay. Expression levels of Akt, ERK1/2, focal adhesion kinase (FAK), Src, Bcl-2, Bax, cytochrome C and cleaved caspase-3 were detected by Western blotting. Integrin β1 mRNA was detected by qRT-PCR. Mitochondrial membrane potential was assayed using a membrane-permeable dye. Hypoxia/SD-induced apoptosis was significantly attenuated by recombinant rat ANGPTL4 in a concentration dependent manner. Moreover, ANGPTL4 decreased the hypoxia/SD-induced caspase-3 cleavage and the cytochrome C release, but increased the Bcl-2/Bax ratio and the mitochondrial membrane potential. Decreased expression of integrin β1, the ANGPTL4 receptor was observed during hypoxia/SD conditions, however, such decrease was reversed by ANGPTL4. In addition, ANGPTL4 induced integrin β1-associated FAK and Src phosphorylation, which was blocked by anti-integrin β1 antibody. ANGPTL4 also reversed the hypoxia/SD-induced decrease of Akt and ERK 1/2 phosphorylation, and the effect of ANGPTL4 was abolished by inhibitors of either integrins, ERK1/2, or phosphatidylinositol 3-kinase (PI3K). Blocking integrinβ1, Akt or ERK largely attenuated anti-apoptotic effect of ANGPTL4. ANGPTL4 protects MSCs from hypoxia/SD-induced apoptosis by interacting with integrins to stimulate FAK complex, leading to downstream ERK1/2 and PI3K/Akt signaling pathways and mimicking the pathway in which MSCs contact with the extracellular matrix.

## Introduction

Despite significant advances in the medical management of heart failure, ischemia/reperfusion injury is still a leading cause of death in developed countries [1]. In the last few years, many investigators have shown that bone marrow-derived mesenchymal stem cells (BM-MSCs) transplantation is a promising tool for both the repair and regeneration of cardiomyocytes and the heart function restoration [2]–[4]. However, the poor survival of engrafted MSCs is a major obstacle in MSC-based therapy. MSCs treatment before transplantation, including treatment with growth factors and cytokines, preconditioning, and genetic modification, has been attempted to enhance the MSCs survival [5]–[7]. Although this pretreatment strategy has proven to be successful in several studies, it showed little benefit to ischemic environment-induced detachment of matrix, and subsequently the apoptotic death of graft cells [8]. Indeed, engrafted MSCs always encounter harsh conditions coupled with the loss of survival signals because of inadequate interactions between cells and matrix [9]. Therefore, enhancement of the anti-apoptotic ability of graft MSCs during the initial settlement to resist apoptosis in harsh conditions and pass survival signals, even in the absence of cell-extracellular matrix (ECM) interaction, would be an attractive approach in development of cell transplantation techniques.

Integrins are cell-surface adhesion receptors composed of α and β subunits, which forms at least 24 heterodimers with different but often overlapping ligands and signaling properties [10]. Signals trafficking via integrins are bidirectional and enable cells to interact with the ECM. Thereby, integrins mediate numerous vital MSCs activities, such as cell shape, adhesion, apoptosis, hypertrophy, survival, differentiation, contraction, and conduction [11]. During cell transplantation, integrins on the donor cells contact with the ECM to initiate survival signaling. However, in an ischemia environment, integrins lose contact with the ECM, lead to apoptosis of the donor cells, and decrease the efficiency of cell transplantation [12]–[14].

Angiopoietin-like 4 (ANGPTL4) was previously identified as a paracrine and, possibly, endocrine regulator of lipid metabolism [15], and as a target of peroxisome proliferators-activated receptors [16]. ANGPTL4 is expressed in numerous cell types, such as adipocytes, cardiomyocytes, and hepatocytes, and is up-regulated after fasting and hypoxia [16], [17]. ANGPTL4 has been found as a strong anti-apoptotic factor in human vascular endothelial cells and colorectal carcinoma cells [18], [19]. It also supports survival of BM hematopoietic stem cells under a serum deprivation (SD) environment [20]. Therefore, it is possible that ANGPTL4 protects engraft MSCs against hypoxia/SD-induced apoptosis.

Recent findings have implicated ANGPTL4 in the regulation of wound healing, tumor cells survival, protection against cardiac infarction, and free fatty acids-induced oxidative stress, in which ANGPTL4 receptors integrins and the associated downstream phosphatidylinositol 3-kinase (PI3K)/Akt (also known as protein kinase B) and extracellular signal-regulated kinase 1/2 (ERK1/2) signaling pathways are also involve in protecting MSCs from apoptosis [12], [13], [21]–[23]. Related to this, recently it has been suggested that ANGPTL4 also plays a role in tumor metastasis by helping tumor cells to resist apoptosis induced by losing contact with the ECM through an integrin-dependent pathway [23]. However, there is no previous report that examines the anti-apoptotic effect of ANGPTL4 in MSCs for regeneration strategies.

We propose that exogenous ANGPTL4 can prevent hypoxia/SD-induced apoptosis of cells, as well as improve subsequent survival of these cells. The present study examined the effect of ANGPTL4 on hypoxia/SD-induced apoptosis of MSCs and its related signal pathways.

## Materials and Methods

### Animals

Male Sprague Dawley (SD) rats weighing 60–80 g were cared for in accordance with US National Institutes of Health published guidelines published by the National Institutes of Health. All of the study procedures were approved by the Harbin Medical University Institutional Animal Care and Use Committee. The study was conducted in compliance with the Guide for the Care and Use of Laboratory Animals published by the National Academy Press (NIH, revised in 1996).

### Reagents

Dulbecco’s modified Eagle’s medium (DMEM) and fetal bovine serum were obtained from HyClone Laboratories (Logan, UT). Trizol reagent was obtained from Invitrogen Corporation (Carlsbad, CA). Transcriptor First Strand cDNA Synthesis Kit and FastStart Universal SYBR Master (ROX) were obtained from Roche (Mannheim, Germany). The Annexin V-fluorescein isothiocyanate (FITC) Apoptosis Detection Kit and anti-CD44, anti-CD29, anti-CD90, and anti-integrin β1 (clone Ha2/5) antibodies were obtained from BD Biosciences (Franklin Lakes, NJ), whereas anti-CD34 and anti-CD45 antibodies were obtained from eBioscience (San Diego, CA). Rabbit monoclonal antibodies, focal adhesion kinase (FAK), Phospho-FAK (Tyr397), Src, Phospho-Src (Tyr-416), Akt, Phospho-Akt (Ser473), Phospho-Akt (Tyr308), Phospho-p44/42 mitogen-activated protein kinase (MAPK) (Thr202/Tyr204, p-ERK1/2), p44/42 MAPK (ERK1/ERK2), caspase-3, Bax, Bcl-2, cytochrome C, LY294002, and U0126 were purchased from Cell Signaling Technology (Danvers, MA). Rabbit monoclonal antibody integrin β1 and rabbit polyclonal antibody ANGPTL4 were obtained from Abcam (Cambridge, UK). Mouse polyclonal antibody β-actin was purchased from Zhongshan Golden Bridge Biotechnology (Beijing, China). Horseradish peroxidase-conjugated secondary antibodies to either mouse or rabbit were obtained from Santa Cruz Biotechnology (Dallas, TX). Alexa Fluor 555 goat anti-rabbit IgG (Invitrogen Technology, USA). ANGPTL4 ELISA kit was obtained from Blue Gene (Shanghai, China). siRNA to ANGPTL4, integrin β1, Akt, and ERK genes were obtained from Life Technologies (Carlsbad, CA, USA). X-treme GENE HP DNA transfection reagent was obtained from Roche (Roche Applied Science, Penzberg, Germany). Recombinant histidine-tagged rat ANGPTL4 (full-length intact form) was obtained from AdipoGen International (San Diego, CA). JC-1 Mitochondrial Membrane Potential Assay Kit was obtained from Beyotine Institute of Biotechnology (Nantong, China). Finally, Cell Counting Kit-8 (CCK-8) assay, Cell Proliferation Assay Kit, was obtained from HaiGene Technology (Harbin, China).

### Cell Culture and Treatment

BM-MSCs were isolated from femurs and tibias of Sprague Dawley rats as described previously by Pittenger *et al.* [24]. Briefly, BM cells were flushed with 5 mL DMEM/F12 from femurs and tibias. After red blood cells were lysed and removed, 5×10^5^ of them were plated in a 25 cm^2^ flask with 6 mL DMEM/F12 supplemented with 10% fetal bovine serum and 1% penicillin/streptomycin at 37°C with a 5% CO_2_ atmosphere. After 3 days of culture, medium and non-adherent MSCs were refreshed with media, while adherent MSCs were further grown in medium, which also was replaced every 3 days. When reaching 80–90% confluence, adherent cells were trypsinized and expanded at either 2∶3 or 1∶2 dilutions. All cells used in the assay were of passages 3 to 5.

MSCs characteristics were demonstrated by immunophenotyping. Cells were harvested, washed with phosphate-buffered saline (PBS), and labeled with the following conjugated antibodies: phycoerythrin-labeled anti-CD45, anti-CD90, FITC-labeled anti-CD44, anti-CD29, and anti-CD34. Labeled cells were analyzed by flow cytometry and with FACSDiva Pro Software (Becton-Dickinson, San Jose, CA).

Induction of apoptosis *in vitro* by hypoxia/SD, designed to mimic the *in vivo* conditions of ischemic myocardium, was initiated as previously described by Zhu *et al.* [25]. Cells exposed to hypoxia/SD alone were used as apoptotic controls. This process was induced by incubating MSCs in serum-free media under a controlled atmosphere (anaerobic chamber), which was generated in a glove box (Plas–Labs, 855-AC) to scavenge free oxygen. Cells cultured in complete medium alone were used as non-ischemic controls.

In preliminary experiments, a time course study involving pre-incubation of cells with ANGPTL4 for 0, 1, and 6 hr was performed, and a 1 hr pre-incubation period was determined as the optimum time point for ANGPTL4 pretreatment prior to exposure to hypoxia/SD. In subsequent studies, ANGPTL4 (100 ng/mL) was initially pre-incubated with MSCs for this time period in complete medium before washing the cells with serum-free DMEM/F12 and re-incubating them in the latter for 24 hr in either the absence or continued presence of ANGPTL4 under hypoxic conditions. In additional control studies, cells were exposed to ANGPTL4 only when they were subjected to hypoxia/SD with no prior pre-incubations. For the optimum concentration, we chose that from 1 to 1000 ng/mL to treat the cells throughout the process.

When used, 25 µM LY294002 (PI3K/Akt inhibitor), 20 µM U0126 (ERK1/2 inhibitor), and 20 µM anti-integrin β1 antibody were pre-incubated with cells in complete medium for a predetermined period of 90 min before exposure to hypoxia/SD, whereas ANGPTL4 (100 ng/mL) was added in the presence of each drug for 1 hr prior to exposure to hypoxia/SD.

### Flow Cytometric Analysis of Cell Apoptosis

Apoptosis was determined by detecting phosphatidylserine exposure on cell plasma membrane with the fluorescent dye Annexin V-FITC Apoptosis Detection Kit, according to manufacturer’s protocols. This assay discriminates intact (Annexin V^−/^propidium iodide -PI^−^), early apoptotic (Annexin V^+^/PI^−^), late apoptotic (Annexin V^+^/PI^+^), and necrotic (Annexin V^−/^PI^+^) cells. Briefly, cells were harvested and washed in ice-cold PBS, resuspended in 300 µL binding buffer, and incubated with 5 µL Annexin V-FITC solution for 30 min at 4°C in dark conditions. This was followed by a further incubation with 5 µL PI for 5 min, and then immediately analyzed by bivariate flow cytometry using the BD FACSCanto II equipped with BD FACSDiva Software (Becton-Dickinson, San Jose, CA). Approximately 1–5×10^5^ cells were analyzed in each sample.

### Terminal Deoxynucleotidyl Transferase-mediated dUTP Nick-end-labeling (TUNEL) Assay

Apoptotic cells were also detected *in situ* by TUNEL assay using an *in situ* Cell Death Detection Kit. The cells for the TUNEL assay were grown on glass coverslips. Cells were fixed for 15 min in 4% paraformaldehyde and the TUNEL reaction was performed according to manufacturer’s instructions. The percentage of DAPI positive and TUNEL positive cells vs. total cells were counted and calculated. At least 1000 MSCs were counted for each dish and averaged. At least three dishes were counted for each group.

### Cell Proliferation Assay

Cell proliferation was assessed by CCK-8 assay according to manufacturer’s protocol. Cells in a 96-well plate were incubated with CCK-8 solutions for 1 hr at 37°C. Absorbance of each well was quantified at 450 nm.

### Toxicity Assay

We tested the ANGPTL4 potential toxicity at different concentrations from cultured MSCs. These cells were incubated with ANGPTL4 in culture medium for 24 hr. According to the material information provided by the manufacture, the compound does not contain bacterial endotoxin or other hazardous substance. Trypan blue was added into the medium, then incubated at 37°C for 15 min before phase contrast graphs were captured by an inverted microscope (Leica DMI4000 B), and trypan blue positive cells were counted. Five fields were randomly selected from each dish, and at least three dishes were counted for each concentration.

### Small Interfering RNA (siRNA) Knockdown

Cells were transfected using the X-treme GENE HP DNA Transfection Reagent, according to the manufacturer’s instructions. In brief, MSCs were plated in a 6-well plate and treated with the X-treme GENE HP DNA Transfection Reagent in a 3∶1 ratio to the siRNA mass for 20 min. Cells were then transfected with a mixture containing 80 mM siRNA and incubated in 2 mL of culture medium for 48 h. Scrambed siRNA (siRNA-NT) was used as the control. Transfection efficiency of siRNA-integrinβ1, siRNA-Akt1, siRNA-ERK and siRNA-ANGPTL4 was analyzed by Western blotting and/or ELISA. The siRNA targeting sequences were listed in Table 1.

**Table 1:** Targeting sequences.

Genes	Sequences
ANGPTL4 siRNA	5′-GCUCUGUGGACUUCAAUCATT-3′
Integrin β1 siRNA	5′-AAAAGTCTTGGAACAGATCTG-3′
Akt siRNA	5′-GAUCUCCUCAUCAUCUGGATT-3′
ERK siRNA	5′-GACCGGAUGUUAACCUUUAUU-3′

### ANGPTL4 ELISA

ANGPTL4 protein was measured in cell culture media using an ELISA kit. The assays were conducted in 96-well microplates according to the manufacturer’s instructions.

### Quantitative Real Time Polymerase Chain Reaction (qRT-PCR)

Expression levels of various genes were analyzed by qRT-PCR. Briefly, total RNAs were isolated and reverse transcribed to cDNA by using the First Stand cDNA Synthesis Kit according to manufacturer’s instructions. qRT-PCR was carried out with FastStart Universal SYBR Master and the ABI fluorescence quantitative PCR system [12]. The threshold cycle (Ct) was set within the PCR exponential phase. The relative gene expression was calculated by comparing cycle times for each target PCR. Target PCR Ct-values were normalized by subtracting the glyceraldehyde-3-phosphate dehydrogenase (GAPDH) Ct-value, which provided the ΔCt-value. The relative expression level between treatments was then calculated using the following equation: relative gene expression = 2^−(ΔCt sample−ΔCt control)^. Primer pairs used to detect messenger RNA (mRNA) levels of target genes were listed in Table 2.

**Table 2:** Primer sequences.

Genes	Sequences
Integrin β1	F: 5′-AAGTGAACAGTGAAGACAT-3′
	R: 5′-CTATCGCAGTTGAAGTTATC-3′
ANGPTL4	F: 5′-GCCGCTACTATCCACTAC-3′
	R: 5′-CCTGTTGCTCTGACTGTT-3′
GAPDH	F: 5′-GGCTCTCTGCTCCTCCCTGTT-3′
	R: 5′-GGCTCTCTGCTCCTCCCTGTT-3′

### Western Blotting Analysis

Western blotting experiments were carried out as previously described by Chen *et al.* [26]. Briefly, cells were washed twice with ice-cold PBS, and then ruptured with lysis buffer containing 20 mM Tris-HCl, 150 mM NaCl, 1% Triton X-100, and protease and phosphatase inhibitors. Cell extracts were centrifuged for 5 min at 12,000×g and supernatants were collected. In all of them, 20 µg cellular protein was resolved by sodium dodecyl sulfate polyacrylamine gel electrophoresis and transferred onto polyvinylidene difluoride membranes. Membranes were blocked for 1 hr with 5% skim milk in Tris-buffered saline containing 0.1% Tween 20, and incubated overnight at 4°C with primary antibodies. Membranes were washed, incubated for 1 hr with appropriate secondary antibodies conjugated to horseradish peroxidase, and developed using chemiluminescence substrates. For its part, membranes were photographed with Bio-Rad ChemiDoc XRS equipment (Hercules, CA), and quantified and analyzed by using the Quantity One software (Bio-Rad, Hercules, CA).

### Immunofluorescence Staining

To investigate the expression of integrin β1 on the surface of MSCs, MSCs were grown on glass coverslips and fixed with 4% paraformaldehyde for 15 min at room temperature, blocked with 10% BSA and incubated with anti-integrin β1 antibody at 4°C over night. After washing, the cells were incubated with the Alexa Fluor 555 conjugated goat anti-rabbit IgG for 1 h at 37°C. The nuclei of cells were counterstained with 49,6-diamidino-2-phenylindole (DAPI). The fluorescence images were acquired with a fluorescence microscope.

### Mitochondrial Membrane Potential (MMP) (ΔΨm) Assay

MMP assay was determined by using the JC-1 Mitochondrial Membrane Potential Assay Kit. Briefly, MSCs were seeded in 6-well plates. After experimental treatment, cells were washed twice with PBS; then 1 mL staining dye/well (culture medium: JC-1 working dye = 1∶1) was added, and cells were incubated at 37°C for 20 min. Cells were washed twice with cold JC-1 staining buffer, and examined under the fluorescence microscope.

### Statistical Analysis

Data were expressed as mean ± SD. Differences among groups were tested by one-way ANOVA, and comparisons between two groups were evaluated using Student’s t-test by using the statistical software SPSS package v19.0 (SPSS, Inc., Chicago, IL, USA). A value of *P*<0.05 was considered as significantly different.

## Results

### MSCs Produced ANGPTL4 upon Exposure to Hypoxia/SD

As a first step, we examined basal ANGPTL4 mRNA expression under hypoxia/SD using qRT-PCR, we confirmed the baseline expression of ANGPTL4 mRNA under hypoxia/SD conditions increased approximately 3 folds compared with the control (Fig. 1A). Moreover, we found that hypoxia/SD stimulated ANGPTL4 release. There was a 2–3 folds increase in release of ANGPTL4 in the medium as compared with the control cells in normoxia (Fig. 1B), in lin with the changes of mRNA level.

**Figure 1:** MSCs produced ANGPTL4 upon exposure to hypoxia/SD. MSCs were cultured under hypoxia/SD or normal conditions for 24 hours. (**A**) mRNA levels of ANGPTL4 molecules were analyzed by qRT-PCR analysis as described in the methods. (Each column represents the mean ± SD of three independent experiments; *P<0.05 vs. control). (**B** ) release of ANGPTL4 was analyzed by ELISA(Each column represents the mean ± SD of three independent experiments; *P<0.05 vs. control).

### ANGPTL4 Protected MSCs from Hypoxia/SD-induced Apoptosis

In preliminary experiments, hypoxia/SD induced MSCs apoptosis with a maximal induction of early apoptosis at 24 hr (Fig. S1). We then examined whether ANGPTL4 could protect MSCs in this process. The data obtained showed a clear anti-apoptotic action of ANGPTL4 (Fig. 2). It was shown that the presence of ANGPTL4 prevented cells undergoing apoptosis, and the most evident protection came from the condition in which cells were pre-incubated with ANGPTL4 for 1 hr prior to the induction of hypoxia/SD, and then continuously incubated with ANGPTL4 for 24 hr (2.63±0.40 vs. 7.48±0.58, *P*<0.05 ) (Fig. 2). Thus, ANGPTL4 was maintained in incubations throughout all following experimental procedures.

**Figure 2:** ANGPTL4 protected MSCs from hypoxia/SD-induced apoptosis. Apoptosis was measured by flow cytometry and TUNEL assay in MSCs pre-incubated with ANGPTL4 (100 ng/mL) for 1 hr, and then either kept (ANGPTL4 Pre-1 hr +24 hr) or removed (ANGPTL4 Pre-1 hr) during a 24 hr hypoxia/SD condition. Cells were exposed to ANGPTL4 when were subjected to hypoxia/SD with no prior-incubations (ANGPTL4 24 hr). MSCs cultured in complete medium were used as controls. (**A and B**) Survival and apoptosis were measured using Annexin V/PI staining and flow cytometry. Annexin V^−/^PI^−^ cells (Q3) were considered as intact or alive cells, Annexin V^+^/PI^−^ (Q4) were considered as early apoptotic cells, Annexin V^+^/PI^+^ cells (Q2) were considered as late apoptotic cells, and Annexin V^−/^PI^+^ cells (Q1) were considered as necrotic cells. One representative experiment out of three is shown in **A**. Quantitative analysis of apoptotic index (fold increase relative to control) by FACS is shown in **B**. (Each column represents the mean ± SD of three independent experiments; *P<0.05 vs. hypoxia/SD; ▴*P*<0.05 vs. ANGPTL4 Pre-1 hr +24 hr). (**C and D**) TUNEL staining on MSCs. The number of TUNEL^+^ cells is shown in **C**. Quantitative analysis of TUNEL^+^ cells (fold increase relative to control) is shown in **D**. (Each column represents the mean ± SD of three independent experiments; *P<0.05 vs. hypoxia/SD; ▴*P*<0.05 vs. ANGPTL4 Pre-1 hr +24 hr).

In further studies, MSCs were exposed to various concentrations of ANGPTL4 (1–1000 ng/mL) followed by exposure to hypoxia/SD for 24 hr. Cell apoptosis was determined by FACS and TUNEL assay (Fig. 3). ANGPTL4 (1–1000 ng/mL) efficiently blocked the apoptotic process as shown by the decreased of TUNEL^+^ cells (Figs. 3B and 3D). The apoptosis degree was also determined by monitoring positivity of Annexin V-FITC stained cells at the end of the incubation period (Figs. 3A and 3C). Exposure of MSCs to hypoxia/SD resulted in a 7.48±0.58-fold increase of Annexin V^+^/PI^−^ cells when compared with controls.

**Figure 3:** ANGPTL4 protected MSCs against hypoxia/SD-induced apoptosis. ANGPTL4 (1–1000 ng/mL) was pre-incubated with the cells for 1 hr in complete medium before exposure to hypoxia/SD conditions, and then was maintained in the incubation medium throughout the hypoxia/SD treatment period. (**A**) Representative image of flow cytometric dot plots analyses of apoptotic cells after Annexin V/PI staining. (**B**) Image showing TUNEL^+^ cells in each group. (**C and D**) Composite values of apoptotic index and percentage of TUNEL^+^ cells. (Each column represents the mean ± SD of three independent experiments; *P<0.05 vs. hypoxia/SD). (**E**) Representative image of Western blots of procaspase-3 cleavage induced by hypoxia/SD and its inhibition by ANGPTL4 using anticaspase-3 antibody. (The blots shown are representative of three independent experiments). (**F**) Composite values of the ratio of cleaved caspase-3 and procaspase-3 relative to β-actin. (Each column represents the mean ± SD of three independent experiments; *P<0.05 vs. hypoxia/SD).

Caspase-3 is one of key mediators of apoptosis, and to further evaluate anti-apoptotic effects of ANGPTL4, we used Western blotting analysis to determine caspase-3 expression. Results showed that ANGPTL4 elicited significant inhibitions of hypoxia/SD-induced caspase-3 cleavage (Figs. 3E and 3F), with the most pronounced effects observed at 100–1000 ng/mL (2.43±0.19 vs. 5.99±0.86, *P*<0.05). However, it was unknown whether ANGPTL4 was toxic to MSCs at these concentrations. Thereby, we examined possible toxicity of ANGPTL4. Trypan blue assay indicated that ANGPTL4 had no adverse effect on the MSCs viability at concentrations up to 1000 ng/mL (Figs. 4A and 4B). It is possible that ANGPTL4 protects cells undergoing apoptosis via promoting the proliferation. Thus, we investigated the effect of ANGPTL4 on cell proliferation. Using the CCK-8 assay, no significant change on cell proliferation rate was found following either a 3-days ANGPTL4 (100 ng/mL) treatment (Fig. 4C) or a 24-hr hypoxia/SD culture (Fig. 4D). Based on these results, all subsequent experiments were performed with 100 ng/mL ANGPTL4.

**Figure 4:** Effects of ANGPTL4 on cell viability and proliferation. ANGPTL4 was added into the culture media alone in order to test its effect on MSCs viability and proliferation. (**A and B**) Trypan blue assessment indicated that ANGPTL4 alone even up to 1000 ng/mL was not toxic to cultured MSCs. (Each column represents the mean ± SD of three independent experiments; *P*>0.05). (**C and D**) Proliferation growth curves of MSCs were obtained by the CCK-8 assay. In the presence of 100 ng/mL ANGPTL4, the proliferation rate did not show significant changes during 3-days ANGPTL4 treatment in the normal culture (**C**), and 24-hr hypoxia/SD culture (**D**). (Each data point represents the mean ± SD of three independent experiments; *P*>0.05).

As above results have confirmed an apparent anti-apoptotic effect of ANGPTL4, we further investigated the effect of knockdown of this gene using siRNA. As shown in Fig.5A to 5C, silencing ANGPTL4 not only largely decreased protein level of ANGPTL4 to 1/3 of control, but also diminished the releasing of ANGPTL4 (6.54±1.10 vs.25.70±4.09, *P*<0.05). At the same time, as shown in Fig.5D and 5E, when the cells exposed to hypoxia/SD, silencing of ANGPTL4 caused more apparent apoptosis than cells only exposed to hypoxia/SD (14.42±1.00 vs.6.53±0.45, *P*<0.05). In contrast, cells transfected with non-targeting siRNA(siRNA-NT) did not show any difference (6.25±0.28 vs. 6.53±0.45, *P*>0.05).

**Figure 5:** Effects of ANGPTL4 on cell survival under hypoxia/SD. MSCs were transfected with a siRNA against the ANGPTL4 transcript. The cells were also transfected witn a non-targeting siRNA(siRNA-NT) as control. The siRNA-mediated transfection efficiency was demonstrated by western blot (**A and B**) and ELISA(**C**). (Each column represents the mean ± SD of three independent experiments; *P<0.05 vs.siRNA-ANGPTL4). Then MSCs were treated with hypoxia/SD for 24 hr. Cells under normal culture were used as control. Then the apoptosis was measured by FACS(**D and E**).(Each column represents the mean ± SD of three independent experiments; *P<0.05 vs. control; ▴*P*<0.05 vs. hypoxia/SD+siRNA-ANGPTL4).

### ANGPTL4 Protected MSCs from Apoptosis through ANGPTL4-integrin β1-related Molecular Pathway

Since integrins mediate numerous vital MSCs activities, we examined if ANGPTL4 protected MSCs from apoptosis through interacting with integrin β1. We evaluated altered expressions of integrin β1 molecules in hypoxia/SD-treated MSCs. As shown in Figure 6A to 6C, the mRNA and protein level of integrin β1 was dramatically increased in ANGPTL4-treated MSCs compared to control MSCs (170.59±9.99% vs.100.00±0.00%, *P*<0.05; 167.54±15.24% vs.100.00±0.00%, *P*<0.05, respectively). Expression of integrin β1 decreased in Hypoxia/SD treated MSCs (28.87±3.63% vs.100.00±0.00%, *P*<0.05; 24.73±3.73% vs.100.00±0.00%, *P*<0.05), however, this decrease was significantly rescued by addition of ANGPTL4 (77.94±9.02% vs. 28.87±3.63%, *P*<0.05; 71.13±6.48% vs.24.73±3.73%, *P*<0.05). Also, the altered expression of integrin β1 was confirmed by immunofluorescent staining. The expression of integrin β1 on the cell surface was increased when treated with ANGPTL4 in a normal condition. Decreased expression of integrin β1 was found in a hypoxia/SD condition, however was rescued by ANGPTL4.

**Figure 6:** ANGPTL4 influenced expression of integrin β1 in MSCs. (**A to C**) mRNA and protein levels of integrin β1 molecules were analyzed by qRT-PCR and western blot analysis as described in the methods. (Each column represents the mean ± SD of three independent experiments; *P<0.05 vs. control; ▴*P*<0.05 vs. hypoxia/SD). (**D**) Expression levels of integrin β1 on the MSCs surfacewere analyzed by immunofluorescence assay.

Integrins are known to activate the cellular FAK and Src at the adhesive stage [27]. In addition, activated integrins bind to the ECM to initiate focal adhesions by recruiting cytoplasmic proteins, such as FAK and Src, which act as linkers between integrins and the actin cytoskeleton to transfer pro-survival signals [28]. Therefore, we investigated FAK and Src expressions. As shown in Figures 7A to 7D, hypoxia/SD treatment significantly decreased the phosphorylation of FAK (21.37±4.62% vs. 100.00±0.00%, *P*<0.05) and Src (21.57±2.41% vs.100.00±0.00%, *P*<0.05) as compared with control MSCs, which were rescued by ANGPTL4 treatment (FAK: 74.43±4.48% vs. 21.37±4.62%, *P*<0.05; Src: 76.03±4.01% vs. 21.57±2.41%, *P*<0.05). Pretreatment of MSCs with anti-integrin β1 antibody abolished the protective effect of ANGPTL4 (FAK: 19.05±3.15% vs. 74.43±4.48%, *P*<0.05; Src: 20.87±3.39% vs. 76.03±4.01%, *P*<0.05) (Figs. 7A–7D).

**Figure 7:** ANGPTL4 protected MSCs from apoptosis through an ANGPTL4-integrin β1 related molecules pathway. (**A to D**) Expression levels of p-FAK (**A and C**) and p-Src (**B and D**) were analyzed by Western blot assay. (Fold changes compared to FAK or Src. Each column represents the mean ± SD of three independent experiments; *P<0.05 vs. control; ▴*P*<0.05 vs. hypoxia/SD+ANGPTL4 ). (**E to H**) MSCs were transfected with a siRNA against the integrin β1 transcript. The cells were also transfected witn a non-targeting siRNA(siRNA-NT) as control. The siRNA-mediated transfection efficiency was demonstrated by western blot (**E and F**). (Each column represents the mean ± SD of three independent experiments; *P<0.05 vs.siRNA-integrinβ1) Then MSCs were treated with hypoxia/SD for 24 hr. In parallel experiments, cells were pretreated with ANGPTL4 (100 ng/mL) 1 hr prior to exposure to hypoxia/SD. The drug was maintained in the incubation medium throughout the hypoxia/SD treatment period. Then the apoptosis was measured by FACS(**G and H**).(Each column represents the mean ± SD of three independent experiments; *P<0.05 vs. control; ▴*P*<0.05 vs. hypoxia/SD, & *P*<0.05 vs. hypoxia/SD +siRNA-integrinβ1).

To further confirm the role of integrin β1 in ANGPTL4 anti-apoptotic effect, we inhibited integrin β1 expression using siRNA, and examined apoptosis of MSCs under a hypoxia/SD condition. As shown in Figure 7E and 7F, siRNA transfection significantly decreased the expression of integrin β1 (40.83±2.95% vs. 100.00±0.00%, *P*<0.05), indicating an effective blocking by siRNA. Siliencing of integrin β1 significantly attenuated the anti-apoptotic effect of ANGPTL4 (6.89±0.30 vs. 3.03±0.18, *P*<0.05). In contrast, no difference was found when transfected with siRNA-NT (2.81±0.32 vs. 3.03±0.18, *P*>0.05).

### ANGPTL4 Protected MSCs from Hypoxia/SD-induced Apoptosis through Integrin-sensitive ERK1/2 and PI3K/Akt Pathways

MAPK and PI3K/Akt signaling pathways have been reported as important regulators in promoting survival of many cells. Therefore, we investigated whether these pathways mediate anti-apoptotic effects of ANGPTL4 in MSCs. Western blotting analysis showed low detectable levels of phospho-ERK1/2 in controls. In contrast, ANGPTL4 induced a pronounced increase in ERK1/2 phosphorylation in a time-dependent manner, with a peak at 60–90 min (4.38±0.34 vs.1.00±0.00, *P*<0.05) (Fig. 8C). Similar to the ERK1/2 phosphorylation, ANGPTL4 also caused a significant increase of Akt phosphorylation in a time-dependent manner, with a peak at 60–90 min [Akt (S473): 4.01±0.66 vs. 1.00±0.00, *P*<0.05; Akt (T308): 4.25±0.43 vs. 1.00±0.00, *P*<0.05)] (Figs. 8A and 8B). Since above data suggested the involvement of both ERK1/2 and PI3K/Akt, we then investigate whether ANGPTL4 protected MSCs from hypoxia/SD-induced apoptosis through integrin β1-sensitive ERK1/2 and PI3K/Akt pathways. As shown in Figures 8D–8F, the Akt and ERK1/2 phosphorylation induced by ANGPTL4 was inhibited not only by inhibitors of these signaling pathways, but also by integrin β1 antibody (20 µM).

**Figure 8:** ANGPTL4 induced ERK1/2 and PI3K/Akt pathways activated. (**A–C**) MSCs were stimulated with ANGPTL4 (100 ng/mL) for the indicated times, and then expressions of Akt and Phospho-Akt (S473) (**A**), Akt and Phospho-Akt (T308) (**B**), and ERK1/2 and Phospho-ERK1/2 (T202/Y204) (**C**) were analyzed by Western blotting. Fold changes were compared to Akt or ERK1/2. (Each column represents the mean ± SD of three independent experiments; *P<0.05 vs. ANGPTL4 −60 min). (**D–F**) Representative image of Western blots of Akt and Phospho-Akt (S473) (**D**), Akt and Phospho-Akt (T308) (**E**), and ERK1/2 and Phospho-ERK1/2 (T202/Y204) (**F**)**.** Under hypoxia/SD, cells that were pretreated with ANGPTL4 (100 ng/mL) and incubated in hypoxia/SD conditions for 24 hr. Compounds on (**D**) and (**E**) were pretreated with LY294002 (25 µM), or integrin β1 antibody. (**F**) was pretreated with U0126 or integrin β1 antibody. Fold changes were compared to Akt or ERK1/2. (Each column represents the mean ± SD of three independent experiments; *P<0.05 vs. control; ▴*P*<0.05 vs. hypoxia/SD+ANGPTL4 −100 ng/mL).

To further confirm the role of PI3K/Akt and MAPK pathways in the anti-apoptotic effect of ANGPTL4, we silenced Akt and ERK using siRNA and examined apoptosis of MSCs under hypoxia/SD conditions. As shown in Figure 9A to 9D, knockdown Akt or ERK genes by siRNA decreased the expression of Akt and ERK to 30.47±5.50% and 20.22±4.33% respectively. Silencing of either Akt or ERK significantly attenuated the anti-apoptotic effect of ANGPTL4 (siRNA-Akt: 7.11±0.40 vs. 3.12±0.29, *P*<0.05; siRNA-ERK: 6.93±0.50 vs. 3.12±0.29, *P*<0.05).(Figure 9E and 9F). In contrast, siRNA-NT did not show significant difference (2.88±0.33 vs. 3.12±0.29, *P*>0.05).

**Figure 9:** ANGPTL4 protected MSCs from Hypoxia/SD-induced apoptosis through integrin-sensitive ERK1/2 and PI3K/Akt pathways. To determine the role of respective kinase pathways in anti-apoptotic actions of ANGPTL4, MSCs were transfected with siRNA against Akt or ERK genes, as well as the scrambled siRNA. The siRNA-mediated transfection efficiency was demonstrated by Western blotting (**A to D**).(Each column represents the mean ± SD of three independent experiments; *P<0.05 vs. siRNA-Akt; *P<0.05 vs. siRNA-ERK). MSCs were then treated with hypoxia/SD for 24 hr. In parallel experiments, cells were pretreated with ANGPTL4 (100 ng/mL) 1 hr prior to exposure to hypoxia/SD, and was maintained in the incubation medium throughout the hypoxia/SD treatment period. The apoptosis rate was analysed by flow cytometry (**E and F**).(Each column represents the mean ± SD of three independent experiments; *P<0.05 vs. control; ▴*P*<0.05 vs. hypoxia/SD+ANGPTL4 −100 ng/mL; &*P*<0.05 vs. hypoxia/SD +siRNA-NT).

### ANGPTL4 Showed Anti-apoptotic Effects via Inhibition of the Mitochondrial Pathway

To examine whether anti-apoptotic effects of ANGPTL4 involve the mitochondrial pathway in hypoxia/SD conditions, we examined the Bcl-2/Bax ratio, the cytochrome C release, the caspase-3 activation, as well as the MMP. ANGPTL4 increased the Bcl-2/Bax ratio (2.70±0.36 vs. 0.34±0.09, *P*<0.05) (Fig. 10A and 10B), and decreased the cytochrome C release (3.00±0.43 vs. 0.48±0.05, *P*<0.05) and the caspase-3 activation (2.72±0.38 vs. 5.70±0.30, *P*<0.05) (Figs. 10C to 10F). In the parallel experiment, ANGPTL4 reversed the decrease of MMP induced by hypoxia/SD (Fig. 10G). The ERK1/2 inhibitor, U0126 (20 µM), the PI3K/Akt inhibitor, LY294002 (25 µM), and the integrin β1 antibody (20 µM), all potently prevented the inhibition caused by ANPTL4 (Fig. 10A–10G).

**Figure 10:** ANGPTL4 exerted anti-apoptotic effects via inhibition of mitochondrial dysfunction. MSCs were treated with hypoxia/SD for 24 hr. In parallel experiments, cells were pretreated with either integrin β1 antibody (20 µM) or LY294002 (25 µM) or U0126 (20 µM) for 90 min before exposure to hypoxia/SD. When present, ANGPTL4 (100 ng/mL) was added in the presence of each drug for 1 hr prior to exposure to hypoxia/SD. All drugs were maintained in the incubation medium throughout the hypoxia/SD treatment period. Bcl-2/Bax ratio (**A and B**), cytochrome C (**C and D**), and caspase-3 (**E and F**) were detected by Western blotting. (Each example shown is representative of three experiments). Fold changes were compared to control. (**G**) MMP with JC-1 staining. (Each column represents the mean ± SD of three independent experiments; *P<0.05 vs. control; ▴*P*<0.05 vs. hypoxia/SD+ANGPTL4 −100 ng/mL).

## Discussion

Autologous MSCs offers a great advantage when used to regenerate and repopulate the injured myocardium, thus restoring heart function after transplantation into ischemic or infarcted heart. Autologous MSCs can be easily prepared from adult patients and they are immunologically safe [29]. However, the MSCs engraftment ratio is extremely low despite large numbers of implanted cells, probably due to a low rate of cell survival induced by the ischemic environment [6], [30]. Despite numerous approaches that have been attempted to overcome these limitations, leading to dramatic improvement of cardiac function in a rodent acute myocardial infarction model, little success has been made to ameliorate the ischemic environment in which MSCs lose contact with the ECM and become apoptotic [31].

Results of the present study suggested that ANGPTL4 effectively protected MSCs from hypoxia/SD-induced apoptosis through the inhibition of mitochondrial dysfunction via integrin-induced PI3K/Akt and ERK1/2 signaling pathways, thus mimicking the signaling pathway induced by cells contacting with the ECM. Thereby, ANGPTL4 may be a good candidate as protective agent to hypoxia/SD-induced apoptosis during cell transplantation and therapy.

ANGPTL4 belongs to a family of angiopoietin-like proteins [32], and is widely identified as a hypoxia-induced gene [33]. In this study, we found that hypoxia/SD condition, which mimicks the *in vivo* ischemic environment, induced the expression and release of ANGPTL4. Furthermore, silencing ANGPTL4 caused large amount of cells undergoing apoptosis in the hypoxia/SD condition, strongly supporting the anti-apoptotic role of ANGPTL4. ANGPTL4 has broad functions and regulates various biological processes, including cell proliferation, migration, angiogenesis, inflammation, and wound healing [22], [33]–[35], although ANGPTL4 was originally thought to participate in glucose and lipid homeostasis [36], [37]. These effects of ANGPTL4 depend on its interaction with receptors, one of these being the integrin β1. During apoptosis, ANGPTL4 interacts with integrin β1 to introduce survival signaling, thus mimicking the signaling introduced by cell-ECM interaction [23]. Moreover, recent studies have demonstrated that integrin β1 takes place in MSCs, and protects these cells from apoptosis when it contacts with ECM [12], [13]. In this study, we found that integrin β1 was expressed on MSCs and increased when treated ANGPTL4, decreased in hypoxia/SD conditions, while was reversed by ANGPTL4. We also found that anti-apoptosis effects of ANGPTL4 were inhibited by the silencing integrin β1. These results strongly suggested that ANGPTL4 protected MSCs from hypoxia/SD-induced apoptosis through an integrin β1-dependent pathway.

Integrins play an important role in mediating the adhesion of cells to the ECM, as well as in regulation of intracellular signaling pathways, which control cytoskeletal organization and cell regeneration and survival. Activated integrins bind to the ECM, cluster at the binding site, and initiate focal adhesions by recruiting cytoplasmic proteins, such as FAK, Src, and paxillin, in order to transfer survival signaling [38], [39]. In this study, integrinβ1 expressed on the surface of MSCs, increased when treated with ANGPTL4. Also, ANGPTL4 up-regulated the FAK/Src complex formation and increased the expressions of phosphorylated FAK and Src, which were abolished by integrin β1 antibody. These results were in line with previous studies, in which integrin β1-dependent signaling stimulated FAK/Src complex formation, in turn activated by contacting the ECM to pass survival signaling [27], [40].

Recent studies have shown that ANGPTL4/ANGPTL4 receptor interaction was associated with an enhanced signaling, regulating levels of phosphorylated Akt and ERK1/2, which regulate various cell functions, such as angiogenesis, immigration, and survival [23], [41], [42]. Since many studies have confirmed an important role of integrin β1-mediated PI3K/Akt and ERK1/2 signaling pathways in cell protection under various conditions, we speculate that integrin β1-dependent PI3K/Akt and ERK1/2 signaling pathways are also important to protect MSCs from hypoxia/SD-induced apoptosis. Our results provided strong evidence to support this hypothesis: ANGPTL4 stimulated Akt and ERK1/2 activation. However, these effects were inhibited by the ERK kinase (MEK)/ERK1/2 inhibitor, U0126 (20 µM), or the PI3K inhibitor, LY294002 (25 µM), or the integrin β1 antibody (20 µM). Furthermore, blocking the expression of Akt and ERK using siRNA largely attenuated the anti-apoptotic effect of ANGPTL4, indicating the involvement of these two signaling pathways following ANGPTL4 treatment.

Previous studies have shown that hypoxia/SD-induced apoptosis in MSCs is sensitive to the mitochondrial apoptotic pathway [25]. Herein, we reported that these processes could be prevented by ANGPTL4 as well. ANGPTL4 inhibited hypoxia/SD-induced mitochondria-dependent apoptosis by increasing the Bcl-2/Bax ratio and the MMP, and by decreasing the cytochrome C release and the caspase-3 activation. These effects are likely mediated via integrin β1-dependent pathways involving both ERK1/2 and PI3K, as anti-integrin β1 antibody, U0126, and LY294002 effectively blocked the effect of ANGPTL4 on the mitochondrial apoptotic pathway.

## Conclusions

In conclusion, we found that ANGPTL4 promoted MSCs survival under conditions that mimic those of the ischemic myocardium. It is likely that ANGPTL4 resists mitochondrial pre-apoptotic changes through integrin-dependent ERK1/2 and PI3K signaling pathways, mimicking pathways activated when cells contacting with the ECM. Our findings propose a new way to protect MSCs from apoptosis, have a considerable therapeutic significance and provide the potential of now exploiting ANGPTL4 and MSCs clinically in cardiac regeneration therapies.

## Supporting Information

Figure S1 **Hypoxia/SD-induced apoptosis of MSCs with a maximal induction of early apoptosis was at 24 h.** (A)Apoptosis was measured by flow cytometry in MSCs when they were cultured in hypoxia/SD conditions for 6, 12, and 24 hr. Flow cytometry showed that hypoxia/SD-induced apoptosis of MSCs with a maximal induction of early apoptosis was at 24 hr. (B) Each column represents the mean ± SD of three independent experiments; ▴*P*<0.05 vs. control; *P<0.05 vs. hypoxia/SD 24 hr.
(TIF)
